# Biomechanical Analysis and Training Method Research on Head Shot Strength of Football Players

**DOI:** 10.1155/2022/7594124

**Published:** 2022-03-15

**Authors:** Yipeng Yao, Shanshan Xiang

**Affiliations:** ^1^Guilin University of Aerospace Technology, Guilin, Guangxi, China; ^2^Guangxi Normal University, Guilin, Guangxi, China

## Abstract

With the development of intelligent sports in China and the rapid improvement of the strength of colleges and universities, the reform of traditional football players' header shooting training methods is becoming more and more urgent in order to solve some problems in the development of sports and speed up the intelligent training of Chinese football players. Based on this, this paper studies the biomechanical analysis and training method based on the integration of header strength data of football players. A dynamic header tracking model of football players based on a local search algorithm is designed. The data collection is realized from the aspects of athletes' header shooting training, skill improvement, physical consumption, and trajectory. The biological data of header shooting power is comprehensively analyzed and evaluated by using a local search algorithm. The results show that the training system based on a local search algorithm has the advantages of high feasibility, high data accuracy, and fast response speed. It can effectively conduct accurate guidance and improve the shooting accuracy according to the biological characteristics of header shooting intensity. This paper studies the biological analysis and training method of header strength of football players based on a local search algorithm. This has certain reference significance for accelerating the construction of intelligent training of Chinese football players.

## 1. Introduction

Up to now, the teaching process of College Physical Education in China is mainly based on the traditional collective and group teaching, supplemented by the independent teaching of the main team members [1]. Since the reform and opening up, the rapid development of various information technologies in China has also led to the reform of China's football system and training methods. The emergence of modern football teaching methods such as team cooperation provides an opportunity for the large-scale development of new football courses in colleges and universities. Intelligence has become an important feature of China's current football training system [2]. At present, although the existing football training system provides a large number of football training methods, it is difficult for players to choose targeted football header shooting training methods according to their own strength structure and biological characteristics in the training process of header shooting and can not achieve the optimal football actual combat effect [3]. In this context, this paper studies the strength characteristics and biological characteristics of the headshot process of government and enterprise players and proposes a dynamic tracking training method of headshot based on the integration of football players' strength information.

The innovation of this paper is to propose a local search algorithm. On this basis, it can make full use of each player's strength training and biological energy characteristic information. Through real-time dynamic tracking, it can achieve the overall approach and quantitatively describe the degree of similarity between the comparison column and the reference column and the degree of agreement between the expected indicators with local correlation factors. By using quantitative indicators to complete the influence degree ranking of training system indicators, it can efficiently carry out customized analysis on the factors affecting players' skill level.

This paper studies the biological analysis of the headshot strength of football players and the construction of training methods, which is mainly divided into three parts. The first part introduces the research status of football training factors at home and abroad. In the second part, the dynamic tracking training model of football player's header shooting based on a local search algorithm is constructed, and the Laplace factor method is used to construct the evaluation index system of header shooting accuracy. The third part tests the evaluation index of the dynamic tracking training system of football players' heading and shooting strength and draws a conclusion.

## 2. Related Work

Since entering the twenty-first century, the training of sports players has encountered difficulties, especially in the construction of football teaching and training systems [4]. Columbia University scholars found that most football training still follows the traditional football training ideas, ignoring the cultivation of practical skills and comprehensive ability. Football training is mainly divided by basic football knowledge, basic football skills and professional knowledge, and broad football skills. Players are not interested in traditional football training. Scholars from Tokyo University of Japan teach according to the rules of football playing and put forward that we should pay attention to the development of classroom-based explanation or teaching video playback, strengthen the development and construction of professional football knowledge courses, and enhance the cognition and attention to football teaching, and the cultivation of football teachers' ability should be improved [5]. According to the multifactor relationship theory and local cooperation theory, a new multirelationship recommendation algorithm is proposed by scholars of Harvard University in the United States, The local weak relation recommendation algorithm has better heterogeneous information acquisition ability than the classical recommendation algorithm [6]. Scholars from Beijing Sport University of China adopted the local search algorithm based on multilocal high weight correlation factors, selected three characteristic parameters related to football players and training system influence indicators, and proposed a dynamic tracking training system for football players' heading and shooting based on local search algorithm for athletes' training characteristic parameters. Football training and other related theories improve the particle swarm optimization algorithm, construct the particle swarm optimization algorithm based on the traditional football training system, and explain the theoretical basis and practical significance of these changes in the algorithm performance with the theory of game theory. Experiments show that the improved algorithm has good local optimization performance [7]. Based on the kinematic theory, scholars from the University of London proposed a hierarchical football header shooting training method. Through the research and analysis of the dynamic differences of weight, height, body fat, and running speed of different football members, it is found that the algorithm can realize the personalized training improvement of hierarchical football players [8]. In order to improve the training efficiency and overall team coordination of football players, scholars from the University of Melbourne in Australia proposed a new team fusion intensive training system based on hyperchaotic mapping through the research of daily training, heading posture analysis and detection, and physical consumption, It is suitable for the analysis of football training and looking for the problems existing in training [9]. Scholars from the University of Toronto in Canada scramble the original football training method by using the transformed chaotic sequence. The results show that the innovative training system has a good overall coordination effect and can resist attack and defense. It can be used in the construction of a football training system [10]. Scholars from Waseda University in Japan proposed a new hyperchaotic cellular neural network football training algorithm to generate the keystream in the team defense stage of football training. The results show that, compared with other related algorithms, this algorithm has the advantages of key sensitivity and strong antiattack and is suitable for football training [11]. Based on the traditional football training fusion strategy technology, scholars from the University of California proposed a panoramic video football cross-border folding search algorithm, which clearly defined the hierarchical framework and index relationship of the whole football training system. This paper evaluates the system from multiple perspectives and provides a comprehensive index sample for the evaluation of the training system of intelligent Chinese football players. Then, it uses the local search algorithm to analyze the characteristics of the players' training results. The results show that the algorithm can effectively reduce the error of football search matching blocks and improve the training efficiency. It is conducive to improving the training skills of heading and shooting in football [12]. Scholars from the Northwestern University of the United States put forward the Fourier function algorithm, and the results show that the algorithm can effectively remove the inefficient cooperation events in the football training system [13]. In order to solve the problem of efficiency and tactical effectiveness of group training, scholars from Shanghai Jiaotong University of China proposed a football competition tactical method based on genetic algorithm and particle swarm optimization algorithm. Experiments show that the algorithm can effectively improve the practicability of football tactics [14]. Scholars from the Hong Kong Polytechnic University of China have realized the tactical evaluation basis in football training by simulating the “modeling structure diagram” in the process of football modeling and improved the flexible transformation from traditional football tactics to modern tactics [15].

To sum up, it can be seen that most of the current football training modes do not involve intelligent depth mining analysis and local search algorithms based on the dynamic training data of football players' heading and shooting. On the other hand, although China has done a lot of basic research, the specific quantitative dynamic evaluation of football intelligent training system and the improvement of football training effect research results are relatively less, and there is no research and related model construction on the intelligence of Chinese football players' heading and shooting training system.

## 3. Methodology

### 3.1. Application Principle of Local Search Algorithm in the Biomechanical Analysis Model of Heading Shot

In order to more intelligently and accurately analyze the specific effect of the signal processing link in the football header shooting, this paper uses the local search algorithm to detect and analyze the head dynamic signal of the football group in the daily football training process. The basic principle of the common local search algorithm is shown in Figure 1, in which DC is the search center.

In this study, the local search algorithm is to find the groups with high similarity of force signals in the process of header shooting from each football player and cluster them. Therefore, the probability of the standard motion data being selected for secondary or multiple detection and analysis is high. On the contrary, if the signal form with a low correlation of dynamic strength structure of football players is selected for secondary or multiple analysis, the probability will be very low. After many times of comparative analyses, the new generation of people with overlapping head ball posture features not only inherits the dynamic head data information of the previous round of intelligent screening but also has a better optimization degree than the information set of the previous generation of eliminated football signals. In this way, after several interactive cycles of two-way heading posture information, the specific information that meets the heading posture requirement conditions corresponding to the lowest normal football skills is finally generated; that is, the analysis value of the normal boundary of a certain football heading posture signal approximates the normal requirement value of the actual heading posture signal. In this way, we can analyze and record the unique heading posture information under the condition of “optimized local search algorithm,” and the mode can also realize the function of self-storage and prediction. The more the process of accumulating the dynamic data of football players' heads, the stronger the self-learning ability and self-evaluation of the system. In addition, in the process of establishing this model, we found that, in the current Chinese long-term football and power sports groups, the analysis of most of the shooting posture of the head ball is based on the traditional detection equipment, and the detection process is mainly direct contact detection. However, noncontact real-time head ball attitude signal detection is rare. Therefore, in this model, a standard structure data evaluation model of football header shooting posture is set in advance (in order to determine the key detection nodes). Therefore, this paper studies the processing object based on the head ball poses randomly selected from the local multigroup head ball pose set of multiple targets to be detected. By comparing with the big data system of the real-time heading posture analysis model of football players, it is very easy to know through simulation that in the two groups with low similarity in the structure of heading posture, it is found that there is a great difference in the skill of shooting between them. And engaged in the football game, the difference in the way of attack will be relatively large.

The above is the basic principle of the local search algorithm used in the research of dynamic signal tracking and data processing of football players' headshots. Through the above optimized local search algorithm, the analysis process is shown in Figure 2, where BN is the connection center, and the rest (*a*, *b*, *c*, *d*, *e*, *f*, *g*, *h*, *i*, *k*) are the classification subcenters. Compared with the common head posture analysis method of football players, it can achieve more accurate analysis and strength correction, which plays a more effective role in the training process of football players' heading and shooting.

### 3.2. Implementation Steps of the Dynamic Tracking Training Model for Football Players' Heading and Shooting

In order to reduce the error analysis of the dynamic signal processing in the training process, we use the local search algorithm with adaptive characteristics. Aiming at the head ball posture signal analysis model of football players in the daily training process, firstly, we will use the big data information and intelligent analysis and processing of the heading posture corresponding to the existing skillful football movements to obtain the initial weight and the minimum threshold value of the heading posture requirement of normal football movement required in the optimized local search algorithm. Then, the local search algorithm is used to analyze and trace the demand degree of heading posture in accordance with the standard with secondary subdivision in the category group of a specific football player's heading posture information. Finally, the optimal solution is searched, and then the real-time dynamic range of heading posture data in the training process is screened out. The three simulation analysis results of the local search algorithm (TSBN, TSFA, and GCSA) are shown in Figure 3, where the horizontal axis is the amount of data and the vertical axis is the cycle index factor.

In the later simulation analysis process, we found that the effect of the traditional local search algorithm is not particularly good. Therefore, in order to improve the detection and intelligent analysis of the head dynamic signal in the football group through the local search algorithm, we need to optimize the local search algorithm, so we use the partial implementation process. In this process, the local search algorithm aims at the dynamic structure of the head ball and the realization process characteristics of the football movement analysis, which is based on the head ball posture information characteristics of the whole crowd target to carry out fuzzy random selection. The purpose of this fuzzy random selection process is to make the signal detection of the common heading posture of different football players more effective because the well-known local search algorithm is not based on a single target in a certain type of feature detection node of the overall target. But through the whole local group of football head ball posture of joint node structure type group to find and get the type of football head dynamic data detection and analysis, the value of the processing conforms to the standard value of the optimal data target. In the process of simulation, the headshot of a random group is taken as the control simulation object. At the beginning of the simulation, the competitive level of one group is lower than the average (the accuracy of the headshot is low), and the other group is lower than the average (the accuracy of the headshot is high). Through nearly 1000 times of simulation experiments and data training under the dynamic tracking model of football players' header shots based on a local search algorithm, it is found that the two groups of data have a great improvement in the comprehensive performance of the new football header shot strength analysis. Therefore, according to the simulation results, the head movement state and strength biological analysis model of the football player has a high accuracy when he is heading, which also shows that the model has good reliability.

Next, the implementation steps and results of the head dynamic signal processing model of football players in the process of training are shown in Figure 4 (under the three methods of TSBN, TSFA and GCSA, the horizontal axis is the amount of data, and the vertical axis is the cycle index factor).

### 3.3. Mathematical Algorithm of the Dynamic Tracking Training Model for Football Player's Headshot

The mathematical operation process is as follows when the dynamic tracking training model of a football player's headshot is realized. First, we need to initialize the parameters. First, let the initial parameter *x*=0 set its judgment function as

(1) $$\begin{array}{c} F_{ij}\left(x\right)=\cos\frac{Nx}{x+1}, \end{array}$$

where *N* is a constant, and *F*_00_(*x*)=0.

Next, the mathematical operation judgment process is verified, and the verification function is

(2) $$\begin{array}{c} H\left(x\right)=\sqrt{\left|\cos\frac{Nx}{x+1}-\sin\frac{Nx}{x+1}\right|}, \end{array}$$

where *N* is a constant and *x* is the amount of information.

We also need to judge the constraints [16]. After the completion of the header shooting data information update, if the end condition is met, the constraint judgment and process update are carried out, and the judgment function is

(3) $$\begin{array}{c} Q\left(x\right)=\left|\frac{s-H\left(x\right)}{\left(s+1\right)H\left(x\right)}\right|, \end{array}$$

where *s* is determined by

(4) $$\begin{array}{c} s=\left(1-\rho \right)*H\left(x\right)+\Delta \tau_{ij}. \end{array}$$

Among them, Δ*τ*_*ij*_=∑_*k*=1_^*m*^Δ*τ*_*ij*_^*k*^, where *τ*_*ij*_ is the length of the current global optimal solution.

Finally, after the pheromone update is completed, the pheromone concentration on each side is limited between [*τ*_*ij*min_, *τ*_*ij*max_], to avoid the pheromone on some sides being too large and reduce the pheromone gap on each side of the graph, so as to expand the search space of the solution, so as to complete the biological analysis of the header shot [17].

## 4. Results of Analysis and Discussion

### 4.1. Design Confirmatory Experiment

Based on the analysis of the above local search algorithms, the system compares the head ball attitude information data of the analyzed target in the process of processing the header shot signal of different players according to the optimized local search algorithm and the intelligent analysis mode of big data of real-time header shooting attitude information based on football players, so the multilevel comparative analysis can be realized. Under this model, there are different ways of heading posture of different football players and we need to know how to analyze whether the tested players' head posture conforms to the best degree of relevant football movements. Through the dynamic analysis model of football head posture after optimization based on multiple comparative analyses and screening, first, the signal similarity of the same football player in the dynamic training process is received, the data processing is carried out, and the relevant unique vector group is obtained. Then, the head ball attitude signal evaluation sample data of different football players are obtained. The data of the unique vector group of the specific single soccer head posture are processed uniformly and orthogonalized. Then, through the automatic comparison and analysis system of the head ball posture of normal football sport based on big data level and the intelligent combination mode of automatic two-way information interaction, and then through the detection and fuzzy processing of various header posture data of local football players, the minimum threshold of initialization weight and the prediction of head ball attitude signal data required by the optimized local search algorithm is realized. The parameter indexes are shown in Table 1.

In this verification experiment, in order to find the relationship between the headshot strength signal processing of football players and the spatial position of intelligent head ball posture, so that the analysis of football head ball posture can bring effective influence on the daily training of football players, this study calls on the local search algorithm, through the first screening and multilevel horizontal and vertical analysis and processing. The initialization weight and the actual threshold of the whole sample are optimized. The optimal vector obtained by the local search algorithm is transformed back as the optimal weight of the local search algorithm and the output average of the ball attitude structure data of football. Through the above process, the head ball posture analysis and the prediction of the future heading posture trend of football can be realized. According to the experimental results, we can find that the model can avoid some complicated links and achieve the same analysis effect or better processing effect in the process of real-time header attitude signal processing of football players. In the process of the research and establishment of the analysis model of the soccer players' real-time head gesture signal processing method, this paper establishes a unique fuzzy detection analysis and processing model from the aspect of the construction of the local search algorithm model.

### 4.2. Experimental Results and Analysis of the Analysis Model of Header Shooting Power

The experimental data of the key node signal under the local search algorithm is shown in Table 2.

The experimental results are shown in Figure 5. The horizontal axis is the number of experiments, and the vertical axis is the positive factor.

According to the results of Table 2 and Figure 5, when analyzing the movement process of different header shots in this football header shooting strength analysis model, we can accurately classify them according to the accuracy of shooting and update them according to the way of high shooting success rate, so as to analyze and summarize their internal verification relationship and continuity. Therefore, according to the experimental results, the dynamic signal detection analysis and processing model based on a local search algorithm can have good accuracy and reliability.

The accuracy results of the experimental results of the signals of key nodes under the local search algorithm are shown in Table 2.

The results of this experiment show that the model can compare and analyze the present state of the header shooting attitude of a specific target (football player) according to the information of key detection nodes, and then, we can know whether the skill of a target in football players is affected by the head ball posture. Therefore, the new method of dynamic signal processing of football players' headshots based on a local search algorithm can be applied to detect and process the real-time head ball attitude signal of professional football players and can complete the monitoring and data analysis of the athletes' posture and strength with high accuracy.

## 5. Conclusion

In this paper, the local search algorithm based on multiple related factors is used to analyze the header strength of football players. Three characteristic parameters related to header shooting and training system are selected, and a dynamic header shooting tracking training system for football players based on a local search algorithm is proposed. Through the research on the improvement of header shooting posture, header technology, and body consumption of football players, this paper expounds on the hierarchical structure and index relationship of the real-time header posture training system of football players. The local search algorithm and ant colony algorithm are used to analyze the characteristics of the screening results. Compared with the existing training search algorithm system, the training system can make full use of each player's football training and game characteristic information, realize the close combination of players, effectively analyze the factors affecting the player's technical level, and improve the player's football training level. However, this paper only focuses on the construction of a dynamic tracking training system for header shooting of football players, without considering the potential impact and overall cooperation of foreign header shooting. Therefore, the comprehensive analysis and evaluation of the index system need to be further studied.

## Figures and Tables

**Figure 1:** The basic principle of the local search algorithm.

**Figure 2:** Analysis process of the local search algorithm.

**Figure 3:** Three kinds of simulation analysis results of the local search algorithm.

**Figure 4:** The process flow chart of the ant system algorithm.

**Figure 5:** Experimental result.

**Table 1:** Experimental data.

Group	Index 1	Index 2	Index 3	Index 4	Index 5
Test group	0.859	0.863	0.952	0.985	0.966
Control group	0.821	0.845	0.914	0.921	0.922

**Table 2:** Accuracy data of experimental results.

Accuracy	Test 1 (%)	Test 2 (%)	Test 3 (%)	Test 4 (%)	Test 5 (%)
Test group	86.9	88.9	95.8	84.0	93.8
Control group	85.8	85.5	89.9	83.9	91.6

## Data Availability

The data used to support the findings of this study are included within the article.
